The article "Telehealth for COVID-19: A Conceptual Framework" was retracted in 2023. Reason: compromised peer review.

# Telehealth for COVID-19: A Conceptual Framework

**DOI:** 10.1155/2023/3679829

**Published:** 2023-02-07

**Authors:** Waqas Yousaf, Arif Iqbal Umar, Syed Hamad Shirazi, Muhammad Fayaz, Muhammad Assam, Javed Ali Khan, Asad Rasheed, Gulzar Mehmood

**Affiliations:** ^1^Department of CS &IT, Hazara University, Mansehra, Pakistan; ^2^Department of Computer Science, University of Central Asia, Naryn, Kyrgyzstan; ^3^Department of Software Engineering, University of Science and Technology, Bannu 28100, Pakistan; ^4^Department of Computer Science, IQRA National University, Swat Campus 19220, Peshawar, Pakistan

## Abstract

The world has been going through the global crisis of the coronavirus (COVID-19). It is a challenging situation for every country to tackle its healthcare system. COVID-19 spreads through physical contact with COVID-positive patients and causes potential damage to the country's health and economy system. Therefore, to overcome the chance of spreading the disease, the only preventive measure is to maintain social distancing. In this vulnerable situation, virtual resources have been utilized in order to maintain social distance, i.e., the telehealth system has been proposed and developed to access healthcare services remotely and manage people's health conditions. The telehealth system could become a regular part of our healthcare system, and during any calamity or natural disaster, it could be used as an emergency response to deal with the catastrophe. For this purpose, we proposed a conceptual telehealth framework in response to COVID-19. We focused on identifying critical issues concerning the use of telehealth in healthcare setups. Furthermore, the factors influencing the implementation of the telehealth system have been explored in detail. The proposed telehealth system utilizes artificial intelligence and data science to regulate and maintain the system efficiently. Before implementing the telehealth system, it is required that prearrangements be made, such as appropriate funding measures, the skills to know technological usage, training sessions, and staff endorsement. The barriers and influencing factors provided in this article can be helpful for future developments in telehealth systems and for making fruitful progress in fighting pandemics like COVID-19. At the same time, the same approach can be used to save the lives of many frontline workers.

## 1. Introduction

The World Health Organization (WHO) declared the outbreak of a public health emergency an international concern. On March 11, 2020, WHO announced COVID-19 as a global pandemic due to a massive increase in the number of cases worldwide, and it is becoming more hazardous due to changing its previous variant. In the wake of the epidemic, countries worldwide suffer from a lack of health resources. They have been making difficult decisions to keep their health services upbeat and their financial conditions normal. All recent reports regarding the spread of COVID-19 have tilted toward the importance of telehealth services [1–3]. The WHO recognized the precautions for slowing down the transmission, issued directions to limit the person-to-person contact through maintaining social distance, and declared detailed public advice. WHO has been updating travel guidelines and continuously adding updates based on scientific findings. Following these precautions can save people from getting infected.

Telehealth can play a pivotal role by providing healthcare facilities to people to effectively combat the pandemic. The country's senior citizens are already under medical treatment and can be checked easily by healthcare workers without putting their lives at risk. The Telehealth system provides comfortable and secure treatment options to save people from overfilled hospitals [4]. It is essential to benefit from the telehealth system as it provides distanced medical services by keeping an epidemic in its view. Typical telehealth programs can be categorized [5] based on stored information (store and forward) like teledermatology, telepathology, teleradiology, etc., programs for monitoring the systems at home, and real-time expert surveillance systems (hospital-based service).

The primary telemedicine services are:

### 1.1. Remote Sensing

It refers to the follow-up, diagnosis, and provision of the latest telemonitoring services to the patients. It is about monitoring the biological parameters of patients through virtual communication between patients and medical professionals to facilitate coordinated actions. Remote assistance separates telecare from telemonitoring. Tele-monitoring facilitates more patients being quarantined at home and monitored properly. Medical experts, citizens, and patients drive these facilities to play a role in managing the disease. Besides this, the telemonitoring system significantly reduces the number of patients in the hospital and lowers hospitals' burden during COVID. The decline has been possible due to virtual communication between health care workers and patients. Virtual communication decreases person-to-person contact and decreases the transmission rate of infection.

### 1.2. Administrative Management of Patients

This service contains laboratory test requirements, billings, and other various concerns. Telehealth services are not always accessible, but governments can make them available in pandemic situations. Still, the records of laboratory tests are to be maintained and followed by medical specialists for further diagnosing the patients.

### 1.3. Distance Learning Service for Professionals

This special service is an essential part of virtual communication related to the guidelines and evidence for educating health professionals. All professionals must use this service to get the latest knowledge and information regarding telehealth systems. The medical experts can join training and seminars through this service.

### 1.4. Evaluation and Collaborative Research Networks

This service refers to the use of ICTs for sharing and spreading the latest practices for building new knowledge through the active participation of individuals. The public and private sectors may implement it in the healthcare setup to make telehealth effective during the COVID-19 pandemic and tackle emergencies. An effective telehealth system needs to be prioritized to get beneficial results in such harsh times. But implementing the telehealth system may face some barriers. This article aims to capture the big picture of barriers and other influencing factors concerning telehealth systems. Barriers need to be minimized, and influencing factors must be followed for the telehealth system's effective implementation. For this purpose, the article highlights some critical requirements for utilizing the telehealth system in global emergencies and the normal routine of life. Moreover, this article proposes a telehealth framework for the COVID-19 pandemic that can minimize p2p contact.

The structure of the proposed research study is as follows: Section 2 discusses the state-of-the-art related work telehealth system.  Section 3 discusses the existing barriers and factors influencing the telehealth system.  Section 4 discusses the proposed telehealth approach.  Section 5 discusses the implications of the proposed approach.  Section 6 concludes the research approach and discusses the future work.

## 2. Use of Telehealth in Emergencies

The provision of telehealth services during unavoidable circumstances enables paramedic staff to help people efficiently. In the current wave of the COVID-19 pandemic, telehealth can access remote areas for general information, and it can help paramedic staff ascertain the situation of the patient's life better. For this purpose, different chatbots have been developed and devised to offload patient surges at the hospitals [6]. Moreover, Telehealth could play a vital role in diagnosis through video conferences with health professionals. Many applications are already available in the market for connecting patients to health professionals via remote video/audio connections, through which patients can be dealt with quickly and efficiently [7–10]. Innovative research in various fields, especially healthcare technology, has revolutionized the world due to synergies between different research fields for improving human lives [11]. Modern healthcare systems provide better ways to understand the dynamics and transmission of diseases like COVID-19. However, accessing modern technologies in all countries might be challenging.

COVID-19 pandemic is not the first reason that pushed governments and healthcare institutions to have telehealth systems. However, the North Atlantic Treaty Alliance (NATO) formerly deployed a Multinational Telemedicine System in 2000 [12]. Telehealth has helped patients from other countries through satellite linkage and personal portable telemedicine kits after approval of the medical experts [13]. Moreover, in natural disasters such as hurricanes in Harvey and Irma cities, private telemedicine companies provided care and medical help to victims who were relocated from their homes [14]. During the severe acute respiratory syndrome (SARS) pandemic in China in 2003, they explored the telehealth system to overcome the upcoming calamity [15]. Similarly, in Australia, during protracted droughts, telehealth has been used to provide additional mental health services through video conferencing under the banner of the medicare benefits schedule launched by the Australian health department [16]. Also, mental health services were provided to Australians affected by bushfires in 2019. It is time to redesign existing healthcare models and understand the critical requirements of COVID-19 to implement the strategies to ensure telehealth [17]. Despite acknowledging the possible benefits of telehealth, its implementation in emergencies has been inadequate [18–20]. Different telehealth frameworks and techniques have been introduced to improve it worldwide. To assist telehealth during the global pandemic[21], introduced a telehealth design blueprint comprising an intelligent way of managing patient's journeys. It provides a complete framework for the healthcare system. However, it allows unlimited increasing rush in the hospitals. The authors in [22] recently proposed an open-source framework, namely OpenTera, that uses software and robotic designers to manage the telehealth system. It consists of independent modules connected under a single framework. However, to fill the gap in telehealth systems, various other factors can be noticed to ensure the proper implementation of telehealth systems.

## 3. Barriers and Influencing Factors in the Use and Implementation of Telehealth Systems and Facilitation Strategies

### 3.1. Barriers to Implementation of Telehealth System

Telehealth implementation in medical systems has been patchy [23, 24] despite tremendous physical and financial efforts by individuals, institutions, and governments, often resulting in a tiny success. To better ascertain the situation, only one per cent of the specialists provided video consultations to the patients, despite substantial financial incentives for medical experts [25]. Similarly, the USA telehealth system suffered the same problems, and only one per cent of the people residing in rural areas took advantage of the telehealth system. In the USA, similar obstacles are found, like doctors' dispositions and other health-related problems. The doctor's inclination toward nonprovision telehealth services in remote areas is the foremost reason for the limited uptake of telehealth [26]. The most convenient method for healthcare providers is telehealth in emergencies, such as outbreaks of COVID-19 around the globe, where the entire health workforce is required to provide immediate care to patients. On the contrary, relying on telehealth in such an emergency is problematic because the patient's physical examination is also needed in some cases.

To ascertain reasons behind the unwillingness to adopt telehealth [27], researchers referred to it as disruptive [28], called it complex, and above all [29] diverted attention toward clinicians' unwillingness to learn new consulting methods. But the emergency telehealth systems cannot be entirely implemented until and unless doctors adopt telehealth, clinicians and paramedic staff as an effective and applicable solution [26]. It may not show effective results as clinicians and paramedic staff have not gone through telehealth training. Once trained, they may know its applicability, harmlessness, and effectiveness [29, 30].

It will be significant to incorporate telehealth into medical curricula so that future healthcare professionals may realize the importance of telehealth being a legitimate part of the healthcare setup. In the literature, researchers reported some issues in implementing technologies such as telemedicine systems (teleconsultation or eHealth systems in general) in healthcare institutions [31–34], indicating internal resistance (within health institutes) to changing normal work processes to accommodate telehealth in organizations [35, 36]. The international literature also pointed out some economic factors, which are huge barriers. According to a US research study, there are no effective reimbursement models for promoting telehealth [37, 38]. The current study captured a big picture summarizing the barriers to implementing the telehealth system as shown and categorized in Figure 1. Four main barriers have been identified in the proposed study, such as technology, organizational, economic, and human barriers, and have been analysed critically with the current state-of-the-art literature and existing systems. Each identified barrier is elaborated in Figure 1. Global and local health authorities can get enough course of action by minimizing the indicated barriers in telehealth systems to implement them successfully.

### 3.2. Factors Influencing Implementation of Telehealth System

In proper standardization and implementation of telehealth systems, critical factors are identified in various literature and from analyzing existing telehealth systems that significantly facilitate and regulate the fast and straightforward incorporation of telehealth projects into successive clinical practice.  Figure 2 identifies and elaborates on some of the summarised key and influencing factors. Incorporating these factors into the telehealth system can improve its performance and efficiency.

## 4. Proposed Telehealth Framework for COVID-19

In this article, we propose a conceptual telehealth framework for COVID-19. The proposed system uses an artificial intelligence technique for screening suspected patients. The screening process may be done with the help of intelligent questionnaires. With the assistance of questionnaires, it is decided whether a patient needs healthcare guidelines, home isolation, or a connection to a telehealth system. The databank will automatically capture the details from Artificial Intelligence-based questionnaires to study the outcomes scientifically in the future. The telehealth system consists of experts who follow up with the patients via video conferencing to make other decisions about the severity of the disease by discussing and reconfirming symptoms that appear on the patient's body. The patient with low severity will be referred to an online monitoring system (OMS), which may consist of nurses and general practitioners. The isolated patient will be referred to the emergency telehealth consultation unit (ETCU) team if the severity is high. If the patient needs to be examined physically, an emergency call will be given to regional rescue services to hospitalize the patient by following all precautionary measures. The training and monitoring unit will handle the medical updates, seminars, training, and staff monitoring. The focus of the proposed telehealth framework is to minimize barriers by providing effective services. The module-wise details, along with the proposed conceptual framework, are shown in Figure 3.

### 4.1. Module 1: AI-Based Questionnaires

Recently, various countries have established emergency phone numbers to prescreen potential cases of COVID-19. Unfortunately, the patients suffered from inability and waiting time due to the massive volume of callers. Intelligent chatbots can work more effectively to tackle this issue [8]. This module technically prescreens the patients by asking questions regarding health conditions. The machine may ask questions based on the responses to previous questions. The machine learning techniques will be applied to designing a questionnaire to understand the degree of urgency [39]. This module will refer the patient to one of three categories, i.e., (a) healthcare guidelines/health media follow-up, (b) home isolation with precautions, or (c) a consultant's prescriptions. This module will significantly reduce the burden on the telehealth system by automatically identifying patient severity categories.

### 4.2. Module 2: Telehealth System

This module consists of senior medical expert teams that specialize in infectious diseases. This board of doctors will examine the patient's data from previous steps, i.e., did the patient follow health media for some days? Or the patient was quarantined at home with the proper precautions given by module 1, and was the patient referred by a consultant to the telehealth system? After that, the patient would be declared to be of low or high severity by expert doctors regarding infectious diseases. This system shall facilitate the patients quarantined at home by avoiding hospital rush. The board may also refer patients with low severity to an online monitoring unit (OMU) and patients with high severity to an emergency telehealth consultation unit.

### 4.3. Module 3: Online Monitoring System (OMS)

This module will be activated for patients with low severity. Nurses and general practitioners (GPs) will be available to follow up with patients to learn about their medical routines. This module requires high-speed Internet as it needs video conferencing. The OMS may refer the patient to a telehealth system, but if the severity increases, the isolated patient will be regularly followed up by nurses and GPs. This online staff will be responsible for updating patients' data so that medical experts can get help with further diagnoses. The OMS shall categorize the low severity patients to avoid their hospital visits. This module will significantly decrease the rush at the emergency telehealth consultation unit (ETCU).

### 4.4. Module 4: Emergency Telehealth Consultation Unit (ETCU)

This module will be responsible for diagnosing the patients who would have been declared to be of high severity by module 2. With the activation of this module, the patient will be treated on an emergency basis. This module contains experts in registered hospitals to handle the emergency. Facilities like Tele-ICU/CCU Teleradiology and artificial intelligence (AI)-based systems may be utilized to analyze patients' medical images and assist radiologists immediately. This module is significant as it deals with critical situations. If the severity of the patient's condition is very high, it may need to be examined physically. The emergency call will be given to the regional rescue service to pick up the patient by following preventive measures. The patient will be admitted immediately to registered hospitals to continue the diagnosis process.

### 4.5. Module 5: Connected AI Labs

Artificial intelligence can be used to diagnose diseases like COVID-19 [40]. This module will be most vital in the diagnostic process for patients with high severity. High-technology labs based on artificial intelligence that provide medical image analysis facilities will generate meaningful analysis reports. Medical images, i.e., CT scans and X-rays, will be processed to determine diseased areas. Data scientists will prepare the medical image analysis reports. The medical image analysis data of patients will be forwarded to ETCU to assist the experts in making decisions about further diagnosis. For significant scientific studies, the medical data will also be shared with module 7 (Data Bank).

### 4.6. Module 6: Training and Monitoring Unit

This module will engage all the workforce of the system with suitable training sessions. The medical updates, seminars, and training will be held through the training unit, and all the updates regarding the telehealth system will be shown. This module will also minimize organizational and human barriers by arranging motivational training for the whole workforce. The module will also be responsible for the availability of doctors, general practitioners, and nurses by inspecting their status.

### 4.7. Module 7: Data Bank

This module will capture the patient's data to engineer it further. Data scientists will perform the scientific study, i.e., breakthroughs, trend analysis, and future predictions of disease.

## 5. Reimbursement/Compensation to Telehealth

Disbursements of telehealth funds and support for the medical healthcare system are prime reasons for uptake and progression [41]. The limitations of telehealth operations vary from country to country. For instance, the Australian Health Department has focused its funding on providing medical consultation via telehealth only in remote/rural areas of Australia. Likewise, telehealth uptake is becoming more challenging, although it can be impartially implemented in urban areas. For infectious diseases like coronavirus (COVID-19), a higher population density in urban areas is at greater risk than in remote/rural areas. Thus, telehealth's potential cannot be denied. Regardless of whether regions are rural or urban, the provision of telehealth facilities is required in case of emergencies all over the globe. Some countries have started addressing these issues by taking the COVID-19 pandemic into view, such as the USA, which in 2020 passed emergency supplemental funding legislation in the wake of COVID-19, expanded its telehealth network to metropolitan areas, and allowed physicians to provide healthcare facilities to patients living in remote areas [42]. The Australian government took similar steps by allowing general healthcare practitioners to offer telehealth consultations [43].

In a crisis, telehealth testing will prove to be a good approach. It will reveal all the flaws, eliminate the errors, and take corrective measures to continue the workflow process for paramedic staff [44]. Preparation and response strategies have already been modulated globally [45]. Moreover, the NATO multinational telemedicine system has assembled software that fulfils all the technological aspects necessary to interconnect diverse national telemedicine competencies [12]. Policies under referred practices shall suit all stakeholders, including patients, health service providers, funding associations (individual and organizational level), and technicians [46–48]. The World Health Organization, National Centers for Disease Control, and health departments at the country level are spreading awareness to control COVID-19 globally through their websites and social media accounts. Furthermore, referred organizations can effectively spread awareness regarding the telehealth system. They can explain its importance and provide specific recommendations concerning telehealth utilization for their public outreach and for countries and noticeable health departments around the globe. There must be detailed future planning for the telehealth system, including hiring experienced consultants and healthcare staff who can effectively fight against pandemics or natural disasters.

## 6. Conclusion and Future Work

Telehealth could play a potential role during emergencies with modern-day technology. The telehealth system can minimize the risk of disease that spreads through contact. Advancement of technology requires strong economic status, and health departments need committed personnel for effective telehealth practices during pandemic situations. Besides the critical barriers to the successful implementation of telehealth, some solutions exist to combat and overcome these barriers. In this article, we captured a big picture of barriers and influencing factors in the way of telehealth systems by studying and analyzing state-of-the-art literature. Considering these barriers and solutions, we proposed a conceptual telehealth framework for COVID-19. This framework can be implemented immediately in response to this global pandemic. Researchers in the health industry and technician training programs can highlight key factors influencing the telehealth system. The proposed framework significantly overcomes the rush burden on hospitals and can help global countries to plan better telehealth policies.

In the future, we will continue working on this application to provide web-based modules by integrating cloud-based services to fight future epidemic emergencies. Future studies may include integrating various online medical image analyses for predicting the intensity of all variants of COVID-19. Moreover, each module of the proposed system can be improved by adding more special features like face recognition for a rapid perception of the patient's health. There is a big door to improving module 5 (Connected AI Labs), i.e., integrating rapid medical image analysis techniques through web-based services.

## Figures and Tables

**Figure 1:** Main barriers to the implementation of telehealth systems. Interrelated factors are responsible for the successful/unsuccessful implementation of the telehealth system. (a) Incorporating new technology requires skills, up-to-date individuals, security, and protection. (b) Lack of strategies, design, and professional conflicts in the organization. (c) High Cost, nonavailability of funds and risk factors of economic investments. (d) Denial of change, conflict of interests, job insecurity, workload, and skeptical attitude.

**Figure 2:** Factors assisting the development of telehealth system. Streamlined aims, capable leadership, effective cooperation, beneficial strategies, minimal complexities, scientific contribution, professional environment, acceptance of culture, resources, and rigorous evaluation can significantly regulate the implementation of telehealth system in the pandemic situation of Covid-19.

**Figure 3:** Proposed telehealth framework for COVID-19. 1. Aims to know the degree of urgency through artificial intelligence-based questionnaires for treatment according to a, b, and c. 2. The main telehealth system consists of senior medical experts' teams for deciding on other processes. 3. Facilitates the patients declared to be of low severity through online consultation of expert nursing and general practitioners' staff. 4. Responsible for diagnosing patients declared to be of high severity using Tele-ICU/CCU/radiology. 5. Provides quick access to highly technologized artificial intelligence labs to perform real-time medical image analysis and generate annotated reports of patients to assist the medical experts. 6. Organize training and seminars regarding any updates. 7. Study the comprehensive data of patients to generate useful statistics.

## Data Availability

The data supporting the findings of this study are available in the paper.
